# SETDB1 Is Involved in Postembryonic DNA Methylation and Gene Silencing in *Drosophila*

**DOI:** 10.1371/journal.pone.0010581

**Published:** 2010-05-17

**Authors:** Dawei Gou, Monica Rubalcava, Silvia Sauer, Felipe Mora-Bermúdez, Hediye Erdjument-Bromage, Paul Tempst, Elisabeth Kremmer, Frank Sauer

**Affiliations:** 1 Department of Biochemistry, University of California Riverside, Riverside, California, United States of America; 2 Zentrum für Molekulare Biologie der Universität Heidelberg, Universität Heidelberg, Heidelberg, Germany; 3 Molecular Biology Program, Memorial Sloan Kettering Cancer Center, New York, New York, United States of America; 4 Institute of Molecular Immunology, Helmholtz Zentrum München, German Research Center for Environmental Health, München, Germany; Radboud University Nijmegen, Netherlands

## Abstract

DNA methylation is fundamental for the stability and activity of genomes. *Drosophila melanogaster* and vertebrates establish a global DNA methylation pattern of their genome during early embryogenesis. Large-scale analyses of DNA methylation patterns have uncovered revealed that DNA methylation patterns are dynamic rather than static and change in a gene-specific fashion during development and in diseased cells. However, the factors and mechanisms involved in dynamic, postembryonic DNA methylation remain unclear. Methylation of lysine 9 in histone H3 (H3-K9) by members of the Su(var)3–9 family of histone methyltransferases (HMTs) triggers embryonic DNA methylation in *Arthropods* and *Chordates*. Here, we demonstrate that *Drosophila* SETDB1 (dSETDB1) can mediate DNA methylation and silencing of genes and retrotransposons. We found that dSETDB1 tri-methylates H3-K9 and binds methylated CpA motifs. Tri-methylation of H3-K9 by dSETDB1 mediates recruitment of DNA methyltransferase 2 (Dnmt2) and Su(var)205, the *Drosophila* ortholog of mammalian “Heterochromatin Protein 1”, to target genes for dSETDB1. By enlisting Dnmt2 and Su(var)205, dSETDB1 triggers DNA methylation and silencing of genes and retrotransposons in *Drosophila* cells. DSETDB1 is involved in postembryonic DNA methylation and silencing of *Rt1b{}* retrotransposons and the tumor suppressor gene *retinoblastoma family protein 1* (*Rb*) in imaginal discs. Collectively, our findings implicate dSETDB1 in postembryonic DNA methylation, provide a model for silencing of the tumor suppressor *Rb*, and uncover a role for cell type-specific DNA methylation in *Drosophila* development.

## Introduction

The enzymatic methylation of position C5 of cytosine in genomic DNA is phylogenetically conserved between prokaryotes and eukaryotes [1]–[2]. In eukaryotes, DNA methylation plays a fundamental role in regulating the structure and activity of DNA and chromatin [3]–[4]. Numerous factors, including DNA methyltransferases (Dnmts), methyl cytosine binding domain (MBD) proteins, chromatin remodeling factors, and enzymes, which support posttranslational modifications of histones (H1, H2A, H2B, H3, and H4), are involved in establishing, maintaining and interpreting DNA methylation [3], [4], [5]. Multiple, intricate DNA methylation machineries mediate and maintain DNA methylation in plants and vertebrates, whereas DNA methylation in *Drosophila melanogaster* (*Drosophila*) appears to involve only an elementary set of factors [5], [6], [7]. One putative Dnmt (Dnmt2) and 5 members of the MBD superfamily of proteins, among them *Drosophila* SETDB1 (dSETDB1) have been identified in *Drosophila* [7]. Dnmt2 mediates DNA and tRNA methylation; silencing of genes, telomers, and transposable elements; as well as methylation of lysine 20 in histone H4 [8], [9], [10]. DSETDB1 is a member of the phylogenetically conserved family of SET/MBD proteins and contains a bifurcated SET domain and an MBD-like domain (MBDL). The SET domain of dSETDB1 methylates lysine 9 in histone H3 [11], [12], [13], [14].

Contrary to the predominant methylation of CpG motifs in vertebrate genomes [15]–[16], The DNA methylation machinery of *Drosophila* preferentially methylates CpA and CpT motifs [17], [18], [19]. The level of DNA methylation is highest in early *Drosophila* embryos, remains detectable in all developmental stages, and decreases in adult flies [17], [18], [19]. In plants, fungi and vertebrates, methylation of H3-K9 by members of the *Su(var)3*–*9* family of histone methyltransferases (HMTs) triggers DNA methylation [20], [21], [22], [23]. In *Drosophila*, Su(var)3–9 mediates DNA methylation during early embryogenesis [9].

The ability of cells to mitotically and meiotically maintain DNA methylation patterns and the low frequency of postembryonic DNA methylation in many organisms supported the model of DNA methylation patterns being static rather than dynamic [3], [24]–[25]. However, the large-scale analyses of DNA methylation patterns in normal and diseased cells and tissues have revealed that DNA methylation is highly dynamic and differentially regulated in response to normal and aberrant intra- and extra-cellular signals [26], [27], [28], [29], [30], [31]. Whether tissue-specific DNA methylation involves DNA de-methylation, as has been suggested for the inactive vertebrate X chromosome [32], or DNA methylation, or both, remains unknown. In addition, how organisms such as *Drosophila* and vertebrates, which establish DNA methylation patterns during the earliest steps of embryogenesis, differentially methylate genes during later stages of development remains unclear [4].

Here, we provide evidence that dSETDB1 is involved in postembryonic DNA methylation and gene silencing in *Drosophila* Schneider 2 (S2) cells and developing imaginal discs. We found that the MBDL of dSETDB1 binds methylated CpA motifs. Methylation of H3-K9 by ectopically expressed dSETDB1 nucleates DNA methylation by Dnmt2 and gene silencing in *Drosophila* cells. In cells and imaginal discs, dSETDB1 cooperates with Dnmt2 and Su(var)205 in DNA methylation and silencing of transposable elements and euchromatic genes such as the tumor suppressor gene *retinoblastoma family protein 1* (*Rb*). Ectopically expressed dSETDB1 propagates the spreading of methylated H3-K9 and DNA methylation on the *Rb* locus in S2 cells, which culminates in the formation of heterochromatin and silencing of *Rb*. Our results implicate dSETDB1 in DNA methylation and gene silencing and uncover a role for DNA methylation in postembryonic development of *Drosophila*.

## Results

### Trimethylation of H3-K9 by dSETDB1 mediates gene silencing

The presence of an MBDL and the described H3-K9-specific HMT activity supports the hypothesis of dSETDB1 being functionally linked to the *Drosophila* DNA methylation machinery [11], [12], [13], [14]. To test this hypothesis, we dissected the role and interplay of the SET domain and MBDL of dSETDB1 in DNA methylation and gene expression. First, we revisited the substrate specificity of the HMT activity of dSETDB1. DSETDB1 can mono-, di- and/or tri-methylate H3-K9 *in vitro* [12], [13], [14], [33] and differentially methylates H3-K9 in a gene-specific fashion *in vivo*. In HMT assays, dSETDB1 methylated H3-K9 in endogenous, purified mononucleosomes and polynucleosomes but did not significantly methylate non-nucleosomal H3-K9 (Figure 1A,B, and Figure S1). The mutation of histone-residue 775 in dSETDB1 (dSETDB1H775L), which is invariant among SET-domain proteins and part of the adenosine-methionine binding pocket [12], attenuated the HMT activity of dSETDB1 (Figure 1A,B). *In vitro* HMT assays coupled to Edman microsequencing (Figure 1C), mass spectrometry (Figures 1D; Figures S2 and S3), and western blot analysis (Figure 1E; Figure S4) revealed that recombinant dSETDB1 tri-methylates H3-K9 in both mononucleosomes and polynucleosomes. Collectively, our data indicates that dSETDB1 preferentially tri-methylates H3-K9 in nucleosomal H3.

**Figure 1:** DSETDB1 preferentially tri-methylates lysine 9 in nucleosomal H3. (**A**) Schematic representation of dSETDB1 and dSETDB1(H775L), which contains a single amino acid exchange mutation of histidine (H) to leucine (L) at amino acid position 775. Rectangles mark the positions of the methyl cytosine binding (MBD)-like domain (MBDL), Pre-SET domain (Pre), SET-domain (SET), and Post-SET domain (Post). The dark box in the SET domain indicates the peptide insertion present in bifurcated SET domain of dSETDB1. (**B**) Coomassie-blue stained SDS-PAGE gel (left) and corresponding fluorogram (right) of histone methyltransferase (HMT) assays containing polynucleosomes, [^3^H]-S-adenosyl-methionine (SAM), and recombinant, immunopurified Flag-epitope–tagged dSETDB1 (lanes 1,3) or Flag-epitope–tagged dSETDB1(H775L) (lanes 2, 4). Asterisks mark the position of anti-Flag antibody light and heavy chain. (**C**) Microsequencing of radiolabeled nucleosomal H3. Polynucleosomes were incubated with recombinant dSETDB1 in the presence of [^3^H]-SAM. H3 was subjected to Edman degradation, and resulting amino acid fractions were analyzed by scintillation counting. The × axis shows amino acids 1–29 of H3. The y axis shows [^3^H]-labeling of amino acids in decays per minutes (D.p.m.). (**D**) Matrix-assisted laser desorption ionization–time-of-flight (MALDI-TOF) spectra of a high-performance liquid chromatography (HPLC) fraction containing the peptide ^9^K(me_0–3_)STGGKAPR of H3. Polynucleosomes were incubated with Flag-dSETDB1 and SAM. H3 was purified and proteolytically digested with trypsin. The resulting peptides were separated by HPLC. Fraction 4 containing ^9^K(me_0–3_)STGGKAPR was subjected to MALDI-TOF mass spectrometry. The × axis indicates the mass:charge ratio. The y axis indicates the abundance of peptides. The positions and m:z ratios of KSTGGKAPR peptides containing non-methylated lysine 9 in H3 (H3-K9), mono-methylated H3-K9 [(me_1_)H3-K9], di-methylated H3-K9 [(me_2_)H3-K9], and tri-methylated H3-K9 [(me_3_)H3-K9] are indicated. (**E**) Western blot analysis of HMT reactions programmed with recombinant Flag-dSETDB1, polynucleosomes, and SAM. Reaction products were separated by SDS-PAGE, electrophoretically transferred onto PVDF membrane, and probed with antibodies to (me_1_)H3-K9, (me_2_)H3-K9, (me_3_)H3-K9, and H3.

Tri-methylated H3-K9 is one hallmark component of heterochromatin [34]; however, dSETDB1-mediated methylation of H3-K9 has been associated with activation and repression of transcription [13]–[14], [33]. To assess the role of dSETDB1-mediated tri-methylation of H3-K9 in gene expression, we performed transient transfection assays in S2 cells. Because dSETDB1 lacks a “classical” DNA binding domain, we used fusion proteins consisting of dSETDB1 and the DNA binding domain of the bacterial tetracycline repressor (TetR) [35]. TetRdSETDB1 fusion proteins repressed the expression of a chromosomal integrated TetR-dependent reporter gene, whereas the HMT-inactive TetRdSETDB1(H775L) and TetR did not (Figure 2A,B; Figure S5). Chromatin immunoprecipitation (ChIP) assays revealed that recruitment of TetRdSETDB1 but not TetRdSETDB1(H775L) mediated tri-methylation of H3-K9 at the reporter gene, which indicates that dSETDB1-mediated tri-methylation of H3-K9, mediates gene silencing (Figure 2C; Figure S6; Table S1).

**Figure 2:** Methylation of H3-K9 by dSETDB1 mediates transcriptional silencing. (**A**) Western blot analysis detecting dSETDB1 (black triangle) and tetracycline repressor (TetR)–SETDB1 (TetRSETDB1) fusion proteins (open triangle) in S2 cells transiently expressing dSETDB1, TetR, or fusion proteins of TetR with dSETDB1 or dSETDB1(H775L). Forty-eight hours after transfection, total cell extracts were prepared, separated by SDS-PAGE, and electrophoretically transferred onto nitrocellulose membrane for probing with antibody to dSETDB1. (**B**) Schematic representation of luciferase assays with whole-cell extracts prepared from cells described in (A). The *tetO-tk-luc* reporter gene contains *tet operator* (*tetO*) sequences, which are fused to the human *thymidine kinase* (*tk*) promoter driving the expression of *luciferase* (*luc*). The diagram shows the mean values calculated from data from 5 different experiments. Error bars indicate the standard error of the mean (SEM). (**C**) Digital images of ethidium bromide-stained agarose gels showing the reaction products of PCR assays monitoring the presence of the promoter region of the *tetO-tk-luc* reporter gene in DNA pools obtained by chromatin immunoprecipitation (ChIP). Chromatin was isolated from (*tetO-tk-luc*)-S2 cells expressing TetR, TetRdSETDB1, or TetRdSETDB1(H775L) and immunoprecipitated with antibodies to dSETDB1, Su(var)205, Dnmt2, (me_3_)H3-K9, and methylated cytosine (^5m^C), or protein-A agarose (control-A) and protein-G agarose (control-G). Input indicates the amount of target DNA present in 1% of the input chromatin.

### The MBDL of dSETDB1 binds methylated CpA motifs

Differences in the primary sequences of the MBD and MBDL have led to the speculation that MBDL proteins do not bind methylated DNA (^m^DNA) [36]. However, the MBDL of dSETDB1 (dSETDB1-MBDL) contains key amino acid residues (such as arginine 436) that are invariant in MBD proteins and essential for the interaction with ^m^DNA [36] (Figure 3A). To test whether dSETDB1-MBDL binds ^m^DNA, we performed *in vitro* protein–DNA binding assays. In our assay system, the MBD of mouse MeCP2, which preferentially binds methylated CpG motifs, interacted with methylated CpG but not CpA and CpT motifs [37]. This result reveals that our assay system can recapitulate the interaction of MBD proteins with ^m^DNA (Figure S7). In contrast the dSETDB1-MBDL (Figure 3B) preferentially bound DNA containing one (Figure 3C; Table S2) or multiple (Figure 3D; Table S2) methylated CpA motifs (^5m^CpA) and bound methylated CpA motifs in DNA containing one methylated CpA, CpT and CpG motif (Figure S8). DSETDB1-MBDL[R436C], which contains a single amino acid exchange mutation of arginine (R) 436 to cysteine (C) (R436C) (Figure 3A,B), did not bind ^5m^CpA motifs (Figure 3E). Our results reveal that dSETDB1-MBDL binds ^5m^CpA motifs *in vitro* and imply that dSETDB1 interacts with ^m^DNA in *Drosophila* cells.

**Figure 3:** The MBDL of dSETDB1 binds methylated CpA motifs. (**A**) Schematic representation of dSETDB1 and the mutant dSETDB1(R436C), which contains the single amino acid exchange mutation arginine (R) to cysteine (C) at position 436. Rectangles mark the positions of the MBDL, Pre-SET domain (Pre), SET domain (SET), and Post-SET domain (Post). (**B**) Coomassie blue-stained SDS-PAGE gel detecting affinity-purified GST, the fusion protein consisting of GST, the MBDL of dSETDB1 (MBDL), and the GST-MBDL(R436C) [MBDL(R436C)] fusion protein. Recombinant proteins were expressed in *Escherichia coli*, purified with glutathione-agarose and subjected to SDS-PAGE. The positions and relative molecular weights of protein standards are indicated. The arrow marks the position of GST-MBDL and GST-MBDL(R436C), the asterisk the position of GST. The protein samples and amounts shown were used for the binding assays shown in (C-E). (**C**) Autoradiogram of *in vitro* protein–DNA interactions detecting the association of [^32^P]-radiolabeled, non-methylated (-) and methylated (+) DNA oligonucleotides containing 1 symmetrically methylated CpG-, CpA- or CpT motif. After proteins were incubated with DNA, retained DNA was purified, separated on native PAGE, and detected by autoradiography. (**D**) Autoradiogram of *in vitro* protein–DNA interaction assays as described in (C) except that methylated DNA oligonucleotides contained 3 symmetrically methylated CpA-, CpT-, or CpG motifs. (**E**) Autoradiogram of *in vitro* protein–DNA interaction assays as described in (C) except that GST, MBDL, and MBDL(R436C) and a DNA oligonucleotide containing 3 symmetrically methylated CpA motifs [(^5m^CpA)_3_] and the corresponding non-methylated DNA oligonucleotide [(CpA)_3_] were used. (C-E) The arrowhead marks the position of retained, radiolabeled DNA.

### DSETDB1-mediated tri-methylation of H3-K9 promotes DNA methylation

Next, we asked whether dSETDB1 is involved in silencing and DNA methylation in *Drosophila*. We used *in vitro* DNA–protein interaction assays designed to identify ^m^DNA target sequences for dSETDB1. Genomic DNA was isolated from 0–12 h old *Drosophila* embryos, sheared and incubated with dSETDB1-MBDL or dSETDB1-MBDL[R436C]. We obtained several DNA sequences that specifically associated with dSETDB1-MBDL but not dSETDB1-MBDL[R436C] (Figure S9). Among the identified DNA sequences are enhancer regions of the genes *Rb*, *Antennapedia* (*Antp*), and *CG2136*, and 2 copies of the retrotransposon *Rt1b*: *Rt1b{}779* and *Rt1b{}999*. The 5155-bp *Rt1b* retrotransposon encodes for a nucleocapsid protein Gag and reverse transcriptase (RvT) and is present in 60 copies in the genome [38]. *Rb* is the *Drosophila* ortholog of the mammalian *Rb* gene [39]. *Rb* proteins regulate the activity of E2F transcription factors and are key regulators of cell proliferation by controlling the G1 and S phases of the cell cycle [40]. During eye development, silencing of *Rb* in response to oncogenic *Notch* signaling involves DNA methylation [41]. The homeotic gene *Antp* is a member of the *HOX* gene family, which is conserved between *Arthropods* and *Chordates*, and involved in cell fate determination during various stages of development [42]. *CG2316* encodes for a putative ABC transporter membrane protein [43].

Because S2 cells apparently do not express dSETDB1 (Figure S10) and the genome of S2 cells is apparently not methylated [44], we transiently expressed wild type and mutant dSETDB1 proteins in S2 cells to assess whether dSETDB1 is involved in the transcription of identified target genes. *Rb*, *Antp*, and *CG2316* are transcribed in S2 cells (Figure 4A; Figures S11-S12). We detected weak transcription of *Rt1b* retrotransposons in S2 cells, which suggests that *Rt1b{}* retrotransposons are transcriptionally active in S2 cells (Figure 4A; Figures S11-S12). However, because of the large copy number of *Rt1b* retrotransposons in the fly genome, we were unable to discern whether the detected transcripts originate from *Rt1b{}779* and *Rt1b{}999*.

**Figure 4:** DSETDB1-mediated tri-methylation of H3-K9 initiates DNA methylation and silencing. (**A**) Digital images of ethidium bromide-stained agarose gels showing the reaction products of RT-PCR assays monitoring the transcription of *Rb*, *Antp*, *CG2316*, *Rt1b/gag*, *dSETDB1*, *Dnmt2*, Su(var)205 and *actin5C* in total RNA pools isolated from S2 cells, S2 cells transiently expressing GFP (control), and S2 cells co-expressing GFP and dSETDB1, dSETDB1(H775L), or dSETDB1(R436C). (**B**) Digital images of ethidium bromide-stained agarose gels showing the products of PCR assays detecting the dSETDB1 target DNA sequence in *Antp*, *CG2316*, and *Rt1b{}799* (see Figure S9) in DNA pools obtained by ChIP. Chromatin was isolated from cells described in (A) and immunoprecipitated with antibodies and controls as described in Figure 2C. 1% of the chromatin used for ChIP.

Transient, ectopic expression of SETDB1 repressed the transcription of *Rb*, *Antp*, *Rt1b* and *CG2316* transcription in S2 cells, whereas dSETDB1(H775L) and dSETDB1(R436C) did not, which suggests that the SET domain and MBDL are involved in dSETDB1-mediated silencing (Figure 4A; Figures S11-S12; Table S1). Ectopic dSETDB1 expression did not significantly affect Dnmt2 and Su(var)205 transcription, which suggests that dSETDB1 is not involved in regulating Dnmt2 and Su(var)205 transcription (Figure S12).

Next, we used ChIP assays to investigate whether silencing of target genes coincides with recruitment of dSETDB1 and methylation of H3-K9 and DNA. Chromatin was isolated from S2 cells expressing dSETDB1 [dSETDB1 cells] or dSETDB1(H775L) [dSETDB1(H775L) cells] and precipitated with antibodies to dSETDB1 (Figure S12); mono-, di-, and tri-methylated H3-K9 [(me_3_)H3-K9] (Figure S4); methylated cytosine (^5m^C) (Figure S13); and Dnmt2 (Figure S14). In contrast to a recent study, we detected the expression of Dnmt2 in S2 cells (Figure S14) [44]. Immunoprecipitated DNA was purified and analyzed with PCR assays that detected the presence of target DNA in immunoprecipitated DNA pools (Table S1).

DSETDB1, (me_3_)H3-K9, ^5m^C, and Dnmt2 were not detected at the transcriptionally active *Rb Antp*, *CG2316* and *Rt1b{}779* loci (Figure 4A,B; Figures S15-S17) and *Rb* (Figure 5A) in S2 cells, but were present at the silent gene loci in dSETDB1 cells (Figures 4A,B and 5A; Figures S15-S18). Tri- but not mono- and di-methylated H3-K9 was detected at silent target genes (Figure S19). In contrast, we detected dSETDB1 but not (me_3_)H3-K9, Dnmt2, and ^5m^C at the target gene loci in dSETDB1(H775L) cells (Figures 4B,5B; Figures S15-S18). Similarly, recruitment of Dnmt2, DNA methylation, and silencing of the *tetO-tk-luc* reporter gene involved dSETDB1-mediated tri-methylation of H3-K9 (Figure 2C; Figures S6 and S19). These results suggest that tri-methylation of H3-K9 by dSETDB1 can instigate DNA methylation and silencing.

**Figure 5:** DSETDB1-mediated tri-methylation of H3-K9 propagates spreading of DNA methylation and silencing of *Rb*. (**A**) Digital images of ethidium bromide-stained agarose gels showing reaction products for the PDE and Exon-I of *Rb* indicated in (A) in DNA pools obtained by ChIP. Chromatin was isolated from S2 cells transiently expressing GFP (control) and S2 cells co-expressing GFP and dSETDB1, dSETDB1(H775L), or dSETDB1(R436C). Chromatin was immunoprecipitated with antibodies and agarose beads described in Figure 2C. PCR assays detected the PDE, PPE and Exon-I in immunoprecipitated DNA pools. (A,C) Input represents the amount of target DNA present in 1% of the chromatin used for ChIP. (**B**) Digital images of ethidium bromide-stained agarose gels detecting the target DNA sequences for dSETDB1 in *Antp*, *CG2136* and *Rt1b{}779* (see Figure S9) in DNA pools obtained by ChIP. Chromatin was isolated from S2 cells transiently expressing GFP and dSETDB1(R436C). Chromatin was immunoprecipitated with antibodies and agarose beads described in Figure 2C. (**C**) Schematic representation of the *Rb* locus. Boxes mark the position of exons I (Exon-I), II, and VIII. The positions of the promoter distal enhancer element (PDE), promoter proximal enhancer element (PPE), and Exon-I fragments detected in ChIP assays are indicated. (**D**) Digital images of ethidium bromide stained agarose gels showing the reaction products of methylation-sensitive restriction analyses of genomic DNA isolated from cells described in (B). Genomic DNA was isolated, incubated with bovine serum albumin (BSA) (mock), the methylation sensitive restriction endonuclease HpaII, or the methylation-insensitive restriction enzyme MspI. PCR assays monitored the presence of the PDE, Exon-I, and the promoter region of *Peepsqueak* (*Psq*) in treated DNA pools.

### Silencing of *Rb* involves initiation and spreading of DNA methylation and heterochromatin

DSETDB1-MBDL is involved in silencing of target genes (Fig. 4A). We performed ChIP assays to assess the role of the dSETDB1-MBDL in silencing and DNA methylation. Chromatin was isolated from S2 cells expressing dSETDB1(R436C) [dSETDB1(R436C) cells]. DSETDB1, Dnmt2 and methylated H3-K9 and DNA were present at the transcriptionally silent dSETDB1 target genes in dSETDB1(R436C) cells (Figures 5A,B; Figures S18 and S20), which implies that the MBDL is not involved in DNA methylation. How does the MBDL of dSETDB1 silence target gene transcription? In S2 cells, silencing of *Rb* coincides with methylation of DNA and H3-K9 at a promoter distal promoter element (PDE) (Figure 5A-C; Figure S9). In developing eye imaginal discs, silencing of *Rb* coincides with DNA methylation at the PDE, a promoter-proximal enhancer fragment (PPE) and first exon (Exon-I) (Figure 5C) [41], thus raising the possibility that dSETDB1 facilitates the spreading of DNA and H3-K9 methylation from the PDE to the coding region. To test this hypothesis, we used ChIP assays to detect dSETDB1-mediated H3-K9 and DNA methylation patterns on the *Rb* locus. Chromatin was isolated from dSETDB1, dSETDB1(H775L), and dSETDB1(R436C) cells and precipitated with antibodies to dSETDB1, (me_3_)H3-K9, ^5m^C, and Dnmt2. Immunoprecipitated DNA was purified and subjected to PCR assays to detect the presence of the PDE, PPE and promoter in immunoprecipitated DNA pools.

We detected dSETDB1, (me_3_)H3-K9, ^5m^C, and Dnmt2 at the PDE, PPE and Exon-I of *Rb* in dSETDB1 cells (Figure 5A; Fig. S18). In dSETDB1(H775L) cells, only dSETDB1 was detected at the PDE (Figure 5A; Fig. S18). In dSETDB1(R436C) cells, SETDB1, (me_3_)H3-K9, ^5m^C, and Dnmt2 occupied the PDE but not the PPE or Exon-I, which indicates that MBDL mediates the spreading of (me_3_)H3-K9 and ^m^DNA from the PDE to the coding region (Figure 5A; Fig. S18). This model is supported by the results of bisulfite DNA sequencing (Figures S16 and S21) and methylation-sensitive restriction analyses (Figure 5D), which reveal an involvement of the SET domain and MBDL in initiation and spreading, respectively, of DNA methylation at the *Rb* locus.

### DSETDB1 cooperates with Dnmt2 and Su(var)205 in *Rb* silencing

The association of HP1 with H3-K9 is a hallmark of silencing in heterochromatin and euchromatin [34]. The interaction of HP1 and Dnmts in vertebrates raised the possibility that Su(var)205 contributes to *Rb* silencing by recruiting Dnmt2 [45]. In ChIP assays, Su(var)205 was detected at the transcriptionally silent *Antp*, *CG2316*, and *Rt1b{}779* (Figure 4B), the *tetO-tk-luc* reporter (Figure 2C) and *Rb* (Figure 5A). In contrast, Su(var)205 and Dnmt2 were not detected at dSETDB1 target genes in the absence of dSETDB1-mediated methylation of H3-K9, which suggests that the association of Su(var)205 with (me_3_)H3-K9 mediates recruitment of Dnmt2 to *Rb* (Figures 2C, 4B, and 5C). Su(var)205 interacted with Dnmt2 but not dSETDB1 *in vitro* and *in vivo*, which suggests that Su(var)205 is involved in recruiting Dnmt2 to target genes for dSETDB1 (Figure S22). To test this, we asked whether destruction of Dnmt2 and Su(var)205 through RNA interference (RNAi) affects dSETDB1-mediated silencing (Figure S23). Knockdown of Dnmt2 or Su(var)205 attenuated dSETDB1-mediated silencing of *Rb* (Figure 6A,B; Figure S24), *Antp*, *CG2316*, and *Rt1b{}* retrotransposons (Figure 7A; Figure S25). Knockdown of Dnmt2 attenuated DNA methylation of *Rb* (Figure 6C,D; Figures S26-S28), *Antp*, *CG2316*, and *Rtb{}799* (Figure 7B,D; Figures S28-S30), whereas knockdown of Su(var)205 prevented recruitment of Dnmt2 and DNA methylation at the *Rb* locus (Figure 6C, right panel, Figure 6D; Figure S26-28), and the *Antp*, *CG2316*, and *Rtb{}799* loci (Figure 7C; Figure S31). Collectively, these results reveal that dSETDB1 cooperates with Su(var)205 and Dnmt2 in DNA methylation and silencing of genes and *Rt1b{}* retrotransposons.

**Figure 6:** Dnmt2 and Su(var)205 cooperate with dSETDB1 in DNA methylation. (**A**) Digital images of ethidium bromide-stained agarose gels showing reaction products of PCR assays detecting *Rb* transcription in total RNA isolated from S2 cells, S2 cells expressing dSETDB1, and S2 cells transiently expressing dSETDB1 in the presence of small-interfering RNA (siRNA) targeting Dnmt2 (Dnmt2-RNAi) or control RNA targeting human GAPDH (mock-RNAi). (**B**) PCR assays as in (A) except that S2 cells were treated with siRNA targeting Su(var)205 [Su(var)205 RNAi]. (**C**) Digital images of ethidium bromide-stained agarose gels showing the presence of the PDE of *Rb* (Figure 5A) in DNA pools generated by ChIP with chromatin isolated from cells described in (a; left panel) and (b; right panel). Chromatin was immunoprecipitated with the antibodies and controls described in Figure 2C. (**D**) Digital images of ethidium bromide-stained agarose gels showing the reaction products of methylation-sensitive restriction analyses with genomic DNA isolated from cells described in (A,B). Assays were performed as described (Figure 5D). PCR assays detected the presence of PDE (Figure 5B) in treated DNA pools.

**Figure 7:** Dnmt2 and Su(var)205 mediate dSETDB1-dependent DNA methylation and silencing of *Antp, CG2316 and Rt1b{}799*. (**A**) (Left panel) Digital images of ethidium bromide-stained agarose gels showing reaction products of PCR assays detecting *Antp, CG2316, and Rt1b{}* transcription in total RNA isolated from S2 cells, S2 cells expressing dSETDB1, and S2 cells transiently expressing dSETDB1 in the presence of small interfering RNA (siRNA) targeting Dnmt2 (Dnmt2-RNAi) or control siRNA targeting human GAPDH (mock-RNAi). (Right panel) PCR assays as in (A) except that S2 cells were treated with siRNA targeting Su(var)205 [Su(var)205 RNAi]. (**B**) Digital images of ethidium bromide-stained agarose gels detecting the presence of *Antp, CG2316, and Rt1b{}* in DNA pools generated by ChIP with chromatin isolated from cells described in (A; left panel) Chromatin was immunoprecipitated with the antibodies and controls described in Figure 2C (**C**) ChIP assays as described in (C) except that chromatin was isolated from cells described in (A; right panel). (**D**) Digital images of ethidium bromide-stained agarose gels showing the reaction products of methylation-sensitive restriction analyses with genomic DNA isolated from cells described in (A,B). Assays were performed as described (Figure 5D) except that PCR assays detected the presence of *Antp, CG2316, and Rt1b{*'*}* in treated DNA pools.

### DSETDB1-mediated DNA methylation facilitates silencing of *Rb* in the developing eye

In the developing eye imaginal disc, *Rb* is expressed in two stripes flanking the morphogenetic furrow (MF), which progresses in a posterior to anterior direction across the eye imaginal disc and induces photoreceptor cell differentiation [46]. Undifferentiated cells exiting the MF undergo a second round of cell proliferation, which includes a single round of synchronized mitosis (second mitotic wave). *Rb* controls the rate of cell proliferation and differentiation in developing eyes by repressing E2F target gene expression [e.g., proliferating-cell nuclear antigen (PCNA)] and mitosis during the second mitotic wave [47].

To assess whether *s*ilencing of *Rb* involves dSETDB1-mediated DNA methylation in *Drosophila*, we attenuated dSETDB1 expression in developing eye imaginal discs by RNAi using the binary Gal4/UAS system [11]. Eye imaginal discs were isolated from *lz^Gal4^*;*UAS-dSETDB1.IR* third-instar larvae. The Gal4-dependent reporter gene *UAS-dEset1.IR* (for simplicity, termed *UAS-dSETDB1.IR*) [11] transcribes an interfering double-stranded RNA targeting the *dSETDB1* mRNA. The *lz^Gal4^* driver expresses Gal4 in all cells posterior to the MF. Western blot and immunostaining assays indicated that dSETDB1 expression is significantly reduced in *lz^Gal4^*;*UAS-dSETDB1.IR* eye discs (Figure S32).

Knockdown of dSETDB1 resulted in ectopic transcription of *Rb* in cells posterior to the MF (Figure 8A). As observed in imaginal discs expressing constitutively active *Rb* [47], ectopic *Rb* expression (Figure S35) suppressed *PCNA* transcription (Figure 8B; Figure S33) and mitosis during the second mitotic wave (Figure 8C) and resulted in defective eye development, as evidenced by the presence of misshaped and fused ommatidia and lack of bristles (Figure 9A,B). To assess the role of Dnmt2 in *Rb* transcription, we monitored *Rb* and *PCNA* expression in eye imaginal discs lacking Dnmt2 through RNAi. Knockdown of Dnmt2 resulted in ectopic expression of *Rb* in cells posterior to the MF (Figure 8A), repression of PCNA (Figure 8B), and attenuation of mitosis (Figure 8C). Collectively, these results indicate that dSETDB1 and Dnmt2 are involved in *Rb* expression in developing eye imaginal discs

**Figure 8:** dSETDB1 represses *Rb* expression in the developing eye. (**A, B**) *In situ* hybridization assays detecting the transcription of (A) *Rb* and (B) proliferating-cell nuclear antigen (PCNA) in eye imaginal discs prepared from control 3^rd^-instar larvae containing the *lz^Gal4^* driver, the reporter *UAS-dSETDB1.IR* or *UAS-Dnmt2, and lz^Gal4^* with *UAS-dSETDB1.IR* (*lz^Gal4^*;*UAS-dSETDB1.IR*) or *lz^Gal4^* with *UAS-Dnmt2* (*lz^Gal4^*;*UAS-Dnmt2*). (**C**) Immunostaining assays detecting the mitotic marker phosphorylated H3 (serine 10) in eye imaginal discs described in (A,B). The mitotic index is38+3 for *lz^Gal4^* eye discs, 37+4 for *UAS-dSETDB1.IR* discs, 36+2 for *UAS-Dnmt2*, 9+3 for *lz^Gal4^*;*UAS-dSETDB1.IR* and 11+2 for *lz^Gal4^*;*UAS-Dnmt2* discs. (A-C) The white-filled arrowheads mark the position of the morphogenetic furrow (MF). (A) Blue arrowheads indicate areas of ectopic *Rb t*ranscription in the posterior region (rectangle) of eye imaginal discs lacking dSETDB1 or Dnmt2, as compared to controls (see area marked by rectangle in *lz^Gal4^* discs). (B) The rectangle marks the position of the posterior PCNA transcription domain. The transcription of the posterior PCNA domain (rectangle) is reduced in dSETDB1 or Dnmt2 deficient eye imaginal discs as compared to controls. (C) The dark arrowhead marks the position of mitotic cells in the second mitotic wave posterior to the morphogenetic furrow. Note that the number of mitotic cells in regions posterior to the morphogenetic furrow (rectangle) is significantly reduced in eye discs lacking dSETDB1 or Dnmt2 through RNAi.

Next we performed ChIP assays to assess whether dSETDB1-mediated repression of *Rb* involves DNA methylation in imaginal discs. We isolated cell stripes from cross-linked eye imaginal discs with the genotype *lz^Gal4^,* and *UAS-dSETDB1.IR* and *lz^Gal4^;UAS-dSETDB1.*IR. Two cell stripes were isolated: one corresponding to the posterior *Rb* transcription domain (P*Rb*D); the second corresponding to the posterior cells flanking the posterior *Rb* transcription domain [posterior cell stripe (PCS)] (Figure 9C). *Rb* is transcribed in the P*Rb*D of control, *lz^Gal4^, UAS-dSETDB1.IR*, and *lz^Gal4^;UAS-dSETDB1.*IR (Figure 8A). *Rb* is not transcribed in the PCS isolated from *lz^Gal4^* and *UAS-dSETDB1.IR* discs (Figure 8A) but is transcribed in the PCS of *lz^Gal4^;UAS-dSETDB1.*IR discs (Figure 8A). Chromatin was isolated from 20 cell stripes, sheared, and immunoprecipitated with antibodies to dSETDB1, ^5m^C, and Dnmt2.

**Figure 9:** DSETDB1-mediated DNA methylation mediates silencing of *Rb* in the developing eye. (**A**) Scanning electron micrographs showing the adult eye phenotype of *lz^GAl4^*, *UAS-dSETDB1.IR* and *lz^GAL4^*;*UAS-dSETDB1.IR* flies (50-fold magnification). (**B**) Magnification of the areas marked by white rectangles in (A) (1,000-fold total magnification). The arrowhead marks the position of fused ommatidia and the arrow the position of misshaped ommatidia. (**C**) (Top) Digital photograph showing *Rb* transcription in eye imaginal disc. The position of the posterior *Rb* transcription domain (P*Rb*D) and posterior cell stripe (PCS) are indicated. (Bottom) Digital images of ethidium bromide-stained agarose gels detecting the PDE of *Rb* in DNA pools obtained by ChIP. Chromatin was isolated from cell stripes representing the P*Rb*D and the PCS of imaginal discs isolated from third-instar *lz^GAl4^*, *UAS-dSETDB1.IR*, and *lz^GAL4^*;*UAS-dSETDB1.IR* larvae. Chromatin was immunoprecipitated with antibodies to dSETDB1, Dnmt2, ^5m^C or rabbit serum (mock). Input represents the amount of target DNA present in 4% of the chromatin used for ChIP.

DSETDB1, ^5m^C and Dnmt2 were not detected at the transcriptionally active *Rb* promoter in the P*Rb*D from *lz^Gal4^, UAS-dSETDB1.IR*, and *lz^Gal4^;UAS-dSETDB1.*IR discs (Figure 9C; Figure S34). In contrast, dSETDB1, ^5m^C and Dnmt2 were present at the transcriptionally silent *Rb* locus in the PCS from *lz^Gal4^* and *UAS-dSETDB1.IR* discs (Figure 9C; Figure S36). We did not detect dSETDB1, ^5m^C or Dnmt2 in the PCS from *lz^Gal^*;*UAS-dSETDB1.IR*, which lacks dSETDB1 and transcribes *Rb* (Figure 9C; Figure S36). Collectively, the results reveal that dSETDB1-mediated DNA methylation is involved in silencing of *Rb* in the developing eye imaginal disc of *Drosophila*.

### DSETDB1 is involved in DNA methylation and silencing of retrotransposons

Because dSETDB1 mediates silencing of *Rt1b{}* retrotransposons in S2 cells (Figures 4 and 7). To test whether dSETDB1 is involved in silencing of *Rt1b[]* retrotransposons in *Drosophila*, we monitored the transcriptional activity and DNA methylation status of *Rt1b{}* and *HeT-A* retrotransposons in developing wing imaginal discs, which lack dSETDB1 and/or Dnmt2 expression by RNAi [11]. *HeT-A* retrotransposons are integral components of *Drosophila* telomers and silencing of *HeT-A* retrotransposons involves dSETDB1-dependent DNA methylation [10]. Wing imaginal discs were isolated from *Gal4(71B);UAS-dSETDB1.IR;UAS-Dnmt2* and control third-instar larvae. The Gal4-dependent reporter gene *UAS-Dnmt2* transcribes an interfering double-stranded RNA targeting the *Dnmt2* mRNA. The *Gal4(71B)* driver expresses Gal4 ubiquitously in imaginal discs. Knockdown of dSETDB1, Dnmt2, or both, resulted in ectopic transcription *of Rt1b{}* and *HeT-A* retrotransposons in wing imaginal discs (Figure 10A-C; Figure S35).

**Figure 10:** DSETDB1-mediated DNA methylation mediates silencing of *Rt1b{}* and *HeT-A* retrotransposons in the developing wing. (**A**) *In situ* hybridization assays detecting *Rt1b* and *HeT-A* transcription in wing (W), haltere (H), and third-instar leg (L) imaginal discs isolated from third-instar larvae, which ubiquitously express Gal4 [*Gal4(71B)*], contain the reporter construct *USA-Dnmt2* and *UAS-dSETDB1.IR* or lack dSETDB1 [*Gal4(71B);UAS-dSETDB1.IR*], Dnmt2 [*Gal4(71B);USA-Dnmt2*], or both [*Gal4(71B);UAS-dSETDB1.IRGal4(71B);USA-Dnmt2*] by RNAi. (**B,C**) RvT-PCR assays monitoring the transcription of *Rt1b{}* and *HeT-A* retrotransposons in wing imaginal discs described in (A). RNA was isolated from 50 wing discs and reverse transcribed. PCR detected the presence of (A) *Rt1b{}* and (D) *HeT-A* transcription. (**D,E**) Digital images of ethidium bromide-stained agarose gels showing the reaction products of PCR assays detecting the presence of (B) *Rt1b{}* and (E) *HeT-A* in DNA pools generated by ChIP. Chromatin was isolated from *in vivo* cross-linked wing imaginal discs isolated from larvae of the genotype described in (A,D). Chromatin was immunoprecipitated with antibodies to dSETDB1, ^5m^C, Dnmt2, Su(var)205, and rabbit serum (control). Input represents the amount of retrotransposons detectable in 2.5% of the input material. (**F,G**) Digital images of ethidium bromide-stained agarose gels showing the reaction products of methylation-sensitive restriction analyses with genomic DNA isolated from wing imaginal discs described in (A). Genomic DNA was isolated, incubated with bovine serum albumin (BSA) (mock), the methylation-sensitive restriction endonuclease HpaII, or the methylation-insensitive restriction enzyme MspI. PCR assays monitored the presence of the (C) *Rt1b{}* and (F) *HeT-A* in treated DNA pools.

Next, we performed methylation-sensitive restriction analyses and ChIP assays to assess whether dSETDB1-mediated repression of *Rb* involves DNA methylation. Chromatin was isolated from *Gal4(71B);UAS-dSETDB1.IR;UAS-Dnmt2*, *Gal4(71B);UAS-dSETDB1.IR, Gal4(71B);UAS-Dnmt2* and control discs. We detected dSETDB1, ^5m^C, Su(var)205 and Dnmt2 at silent *Rt1b[]* and *HeT-A* retrotransposons. Knockdown of dSETDB1 and/or Dnmt2 resulted in loss of DNA methylation at *Rt1b{}* (Figures 10D,F; 1) and *HeT-*A (Figure 10E,G; Figures S36, and S37; Table S1) retrotransposons, which indicates that dSETDB1-mediated DNA methylation is involved in silencing of *RT1b{}* and *HeT-A* retrotransposons.

## Discussion

Collectively, our results implicate dSETDB1 in postembryonic DNA methylation and silencing of genes and transposons. Despite significant progress, the functional importance of DNA methylation in *Drosophila* remains controversial, and important mechanistic aspects of the DNA methylation process remain unknown [4], [7]–[8]. DSETDB1 is involved in oogenesis, maintenance of heterochromatin, silences gene expression in pericentric heterochromatin, and activates and represses transcription in the peculiar chromatin of the fourth chromosome, respectively [11], [12], [13], [14], [33]. Our results reveal that dSETDB1 is an integral component of the *Drosophila* DNA methylation machinery. The functional dissection of the SET domain and MBDL reveals that dSETDB1 is an epigenetic repressor. The activity of the SET-domain initiates silencing and DNA methylation, whereas the MBDL can facilitate propagation of DNA methylation. DSETDB1 conveys epigenetic silencing by directly and indirectly supporting the placement of 2 epigenetic marks at target genes: (me_3_)H3-K9 and ^m^DNA.

The dSETDB1-MBDL preferentially associates with methylated CpA motifs *in vitro*, which represents one of the two predominantly methylated DNA motifs in the *Drosophila* genome. In *Arabidopsis thaliana*, MBD proteins bind methylated CpG- and CpNG motifs and can associate with ^5m^C in any DNA sequence context [48]. The interaction of dSETDB1-MBDL with methylated CpA motifs suggests that *Drosophila* has evolved specialized factors to translate CpA methylation into biological function. Although the genomes of many *Arthropods* and vertebrates contain methylated CpN motifs and often express multiple MBDL proteins, the biological importance of CpN methylation in development and disease remains mysterious [15], [36], [49]. The association of dSETDB1-MBDL with methylated CpA motifs supports a model for MBDL proteins interpreting complex patterns of CpN methylation into distinct biological activities.

Recent studies revealed that dSETDB1 mono-, di-, and/or tri-methylates H3-K9 [11]–[12]. However, the mechanisms underlying the gene-specific, differential methylation of H3-K9 by dSETDB1 remain unknown. It appears possible that intra- and extra-organismal stimuli modulate the specificity of the catalytic activity of dSETDB1, which results in gene-specific mono-, di- or tri-methylation of H3-K9. Our studies uncover a role for dSETDB1-mediated tri-methylation of H3-K9 in DNA methylation, but do not exclude the possibility that mono- and/or di-methylation of H3-K9 by dSETDB1 might trigger DNA methylation in the context of other genes.

In *Drosophila*, plants, vertebrates, and *Neurospora crassa*, members of the Su(var)3–9 family play pivotal roles in DNA methylation [9], [20], [21], [22], [23]. Su(var)3–9 facilitates DNA methylation during *Drosophila* embryogenesis and is apparently not involved in postembryonic DNA methylation [9]. Because dSETDB1 is not expressed during the early stages of embryogenesis, when global DNA methylation occurs [11], it appears likely that dSETDB1 does not play a major role in embryonic DNA methylation. The involvement of dSETDB1 in DNA methylation and silencing of *Rb* and *Rt1b{}* retrotransposons in imaginal discs suggests that the differential activities of at least 2 distinct HMT pathways mediate embryonic and postembryonic DNA methylation in *Drosophila*: the Su(var)3–9 pathway acting during embryogenesis and dSETDB1 pathway during postembryonic stages. This hypothesis is supported by a recent study by Elgin and colleagues, which revealed that Su(var3–9) activity is restricted to early development, whereas dSETDB1 acts preferentially during later stages of development [33].

The role and function of Dnmt2 in DNA methylation remains controversial [8], [10]. In a recent study, Reuther and colleagues have linked Dnmt2 with DNA methylation at transposable elements and telomers [10]. The observed loss of DNA methylation and silencing of genes and retrotransposons in cells and imaginal discs, which lack Dnmt2 through RNAi supports the role for Dnmt2 in DNA methylation, differential gene expression, and silencing of transposon activity during *Drosophila* development. However, our results do not exclude the possibility that the observed Dnmt2-dependent DNA methylation does not involve the catalytic activity of Dnmt2 but rather other unknown Dnmts, which are recruited to dSETDB1 target genes in a Dnmt2-dependent fashion.

Silencing of retrotransposons is fundamental for the structural integrity of eukaryotic genomes. Our results reveal that dSETDB1 contributes to genome stability by silencing *Rt1b*{} and *HeT-A* retrotransposons. Our results reveal that *Drosophila* uses epigenetic regulators and mechanisms involved in heterochromatin formation to silence the activity of retrotransposons and genes such as the essential cell cycle regulator *Rb* and during development.

The results of transient expression experiments in S2 cells support a model for dSETDB1-mediated silencing of *Rb*: recruitment of dSETDB1 and subsequent methylation of H3-K9 resulted in recruitment of Su(var)205 and Dnmt2 to the PDE and DNA methylation. Because the MBDL can interact with methylated CpA motifs, methylation of CpA motifs may result in *de novo* recruitment of dSETDB1 proteins or allow PDE-associated dSETDB1 to bind ^m^DNA downstream of the PDE. In both cases, recruitment of dSETDB1 triggers a self-perpetuating, self-renewing H3-K9 and DNA methylation cascade, which culminates in the silencing of *Rb*. Similarly, silencing of retrotransposons in *Drosophila* involves propagation of DNA methylation [10].

Why does silencing of *Rb* involve heterochromatin formation at the enhancer, promoter, and coding region? In vertebrates, methylation of promoter-proximal CpG islands has been linked to gene silencing [15]. DNA methylation can silence gene expression by preventing the interaction of transcription factors and the RNA polymerase II transcription machinery with target genes [5], [50]–[51]. However, CpG methylation and CpG islands are rare in *Drosophila* [17], [18], [19]. Thus, in the absence of CpG islands, DNA methylation and subsequent heterochromatin formation at the enhancer, promoter and coding region of *Rb* may be necessary to prevent the association of transcriptional regulators with *Rb* and, consequently, the initiation and elongation steps of transcription.

*Rb* proteins play important roles in development, and the precise temporal and spatial expression of *Rb* is fundamental for cell proliferation and differentiation [40]. Our results suggest that epigenetic silencing of *Rb* during eye development in *Drosophila* involves dSETDB1-mediated DNA methylation and heterochromatin formation. Most cells in metazoan organisms are quiescent [52]. Epigenetic silencing of cell cycle regulators upon completion of development may maintain the quiescent state after completion of cell differentiation and proliferation. DNA methylation and silencing of tumor suppressor genes has been correlated with various human diseases such as cancer [53], [54], [55]. Our results shed new light on the mechanisms involved in DNA methylation and silencing of tumor suppressor genes and provide a foundation for the dissection of the role of SET/MBDL proteins in dynamic DNA methylation during cell proliferation in development and disease.

## Materials and Methods

### Plasmids

Detailed information about the recombinant DNA used in this study can be found in Text S1.

### Chromatin immunoprecipitation (ChIP)

Chromatin immunoprecipitation was performed as described [56]. Cross-linked chromatin was isolated from FACS-sorted *Drosophila melanogaster.* S2 cells expressing wild type or mutant dSETDB1 proteins or TetRdSETDB1 derivatives, and wing imaginal discs and sections of eye imaginal discs, which were isolated from wild type and mutant larvae. Chromatin was immunoprecipitated with antibodies to *anti*-5-methyl cytosine (Megabase, #CP51000), *anti*-(me_3_)H3-K9 (Abcam, ab8898), *anti*-Dnmt2 (this study), *anti*-dSETDB1 (this study), and *anti*- Su(var)205 (this study). A detailed ChIP protocol is available in Text S1.

### Mono- and polyclonal antibodies

The rat monoclonal antibody to dSETDB1 was developed against the peptide K-796-2 NNSTIYVDDENRC (amino acids 351–362). Immunization, fusion, and cloning were performed as described [59]. Polyclonal antibodies against Dnmt2 and Su(var)205 were generated in rabbits with use of the peptides Dnmt2-7A53-2 (amino acids 64–84) and Su(var)205 3C78-2 (amino acids 72–91). Polyclonal antibodies were produced by Biosynthesis (Lewisville, Texas, USA).

### Protein-DNA binding assays

Protein-DNA binding assays were performed as described [37]. GST, GST-MBDL and GST-MBDL(R436C) were expressed in and purified from *Escherichia coli* XL1-Blue (Stratagene). The GST proteins were immobilized on glutathione-sepharose beads (Invitrogen). To reduce unspecific interactions, 100 µl of protein-loaded glutathione-sepharose beads were preincubated with 0.5 µg/µl yeast DNA in 500 µl binding buffer (BB) (25 mM Tris-HCl pH 7.5, 50 mM KCl, 1 mM DTT, 5% [v/v] glycerol) at 4°C for 3 h. An amount of 10 µl of pre-incubated glutathione-sepharose beads loaded with 250–500 ng GST or GST-dSETDB1 derivatives were incubated with [^32^P]-labeled radiolabeled oligonucleotides (150,000 c.p.m./reaction) in BB at 4°C for 4 h. The DNA oligonucleotides were unmethylated or contained 1 or 3 ^m^DNA motifs (Table S2). After incubation, beads were precipitated and washed twice with BB, 4 times with BB containing 500 mM NaCl, and twice with TE. Retained DNA was purified by phenol/chloroform extraction, separated on native polyacrylamide electrophoresis, and detected by autoradiography.

### RNAi

Small interfering RNAs (siRNAs) targeting Su(var)205 and Dnmt2 were designed using the “siRNA at Whitehead” [57] generated by *in vitro* transcription using the silencer siRNA construction kit (Ambion). S2 cells, 5×10^6^, were transfected with 1–4 µg siRNA by use of oligofectamine (Invitrogen) and harvested after 3–5 days. Western blot analyses confirmed destruction of the target protein. A detailed description of the siRNAs used for RNAi is available in Text S1.

### Fly strains

The following fly strains were used: *OregonR* (Bloomington stock center: #5), *12196*–48 [11], *lz^Gal4^* [58] (Bloomington stock center: #6313), gal4(71B) [59] and *actin5C^Gal4^* (Bloomington stock center: #3954). Fly strains were maintained and crossed using standard media and procedures [60].

## Supporting Information

Text S1 Supporting Information: Materials and Methods.
(0.09 MB DOC)

Figure S1 DSETDB1 methylates H3-K9 in nucleosomal H3. Coomassie blue-stained SDS-PAGE gel (left) and corresponding fluorogram (right) of HMT-assays containing a mixture of recombinant histones H2A, H2B, H3, and H4 (H-mix); purified, endogenous mononucleosomes (mono nucl); or purified, endogenous polynucleosomes (poly nucl). Histones were incubated with [^3^H]-SAM) (-), [^3^H]-SAM and “*anti*-Flag antibodies coupled to agarose beads” (“Flag-beads”), which had been incubated with *Sf*9 extract (Flag-beads), or [^3^H]-SAM and Flag-beads, which had been loaded with Flag-tagged, recombinant dSETDB1 (Flag-beads-dSETDB1). Reaction products were separated by SDS-PAGE and detected by fluorography. Asterisks indicate the positions of the *anti*-Flag antibody light and heavy chains.
(3.86 MB EPS)

Figure S2 DSETDB1 methylates H3-K9. (A) MALDI-TOF spectrum of the HPLC fraction containing the peptide ^9^K(me_0–3_)STGGKAPR. Shown is the complete spectrum corresponding to the MALDI-TOF spectrum shown in Fig. 1D. In addition to ^9^K(me_0–3_)STGGKAPR peptides, the HPLC fraction contains two peptides (peptide A, measured mass 573.362; peptide B, measured mass 630.412). The inset represents a magnified area of the spectrum shown in Fig. 1D. The x-axis indicates the mass/charge ratio. The y-axis indicates the abundance of peptides. (B) Table indicating the measured and calculated masses of detected peptides ^9^K(me_0–3_)STGGKAPR. ΔM/M represents the relative errors between measured and calculated masses.
(0.61 MB EPS)

Figure S3 DSETDB1 preferentially tri-methylates H3-K9 (A) Nano-ESI MS/MS spectrum of the spectrum of the precursor ion at m/z 472.28 of peptide ^9^K(me_3_)STGGKAPR, which was obtained from the HPLC fraction shown in Fig. S2. The y-axis indicates abundance of peptides (ion counts), the x-axis represents the mass/charge ratio (m/z). (B) Nano-ESI MS/MS spectrum as in (A) except that the precursor ion at m/z 465.28 of peptide ^9^K(me_2_)STGGKAPR was analyzed. (C) Nano-ESI MS/MS spectrum as in (A) except that the precursor ion at m/z 458.27 of peptide ^9^K(me_1_)STGGKAPR was analyzed. (A-C) The inset shows the fragmentation schematic for the b and y series of the corresponding precursor ion.
(0.64 MB EPS)

Figure S4 Western blot assays testing the specificity of antibodies recognizing mono-, di-, and tri-methylated H3-K9. 2 µg H3 peptides (amino acids 1-40) containing mono-, di- or tri-methylated H3-K9 were separated by SDS-PAGE and electrophoretically transferred onto PVDF. Blots were developed with antibodies to mono-methylated H3-K9 [*anti*-(me_1_)H3-K9; top], di-methylated H3-K9 [*anti*-(me_2_)H3-K9; middle] and tri-methylated H3-K9 [*anti*-(me_3_)H3-K9; bottom].
(1.03 MB EPS)

Figure S5 Basal transcription level of the *luciferase* (*luc*) gene in the stable cell line (*tetO-tk-luc*)-S2. RvT-PCR assays detecting the mRNA of (top) *luc* and (bottom) *actin5C* in total RNA pools isolated from S2 cells and the stable cell line (*tetO-tk-luc*)-S2 cells. Arrowheads indicate the position of the PCR products.
(0.64 MB EPS)

Figure S6 DSETDB1-mediated tri-methylation of H3-K9 mediates repression and DNA methylation. Schematic representation of Real-Time PCR assays corresponding to the conventional PCR assays shown in Figure 2C. RT-PCR assays were performed using the same DNA pools used for conventional PCR. The degree of association of an antigen with the target DNA was calculated as fold enrichment by comparing the number of target DNA molecules in DNA pools obtained in ChIP assays using control antibodies with reactions containing antibodies to specific antigens.
(0.25 MB EPS)

Figure S7 The MBD of MeCP2 binds methylated CpG-motifs. Autoradiogram of DNA-protein interaction assays programmed with DNA oligonucleotides containing one symmetrically methylated CpG-, CpA-, or CpT-motif and recombinant GST or fusion proteins consisting of GST and the MBD of MeCP2. Retained DNA was purified, separated by native PAGE, and detected by autoradiography. The arrowhead marks the position of retained DNA oligonucleotides.
(2.83 MB EPS)

Figure S8 The MBDL of dSETDB1 preferentially binds methylated CpA motifs. (Top) Schematic representation of the 105 bp target DNA fragment C(ATG)-1. The positions of EcoRI restriction sites, the length of the DNA fragments (a,b,c) resulting from EcoRI digest, and the methylated CpN motifs present in fragments a, b, and c are indicated. (Bottom) Autoradiogram of *in vitro* DNA-protein binding assays. The 105 bp target DNA was incubated with glutathione beads loaded with GST, GST-MBDL, or GST-MBDL(R436C) (see Figure 3). Bound DNA was digested and digested with EcoRI. Retained, radiolabeled DNA was eluted. Retained DNA was separated by native PAGE and detected by autoradiography. The positions of radiolabeled DNA fragments (a, b, and c) are indicated.
(0.57 MB EPS)

Figure S9 Identification of target genes for dSETDB1. (A) Digital image of ethidium bromide-stained agarose gel showing the affinity-purified genomic DNA. DNA was isolated from 0-12 h old *Drosophila* embryos and sonicated (input, lane 1). Genomic DNA was sequentially incubated with the MBDL of dSETDB1 (lane 2), the mutant MBDL(R436C) (lane 3), and the MBDL of dSETDB1 (lane 4). Purified DNA was amplified by PCR (lanes 2-3) cloned and sequenced. Input represents 0.1% of the input DNA used for the affinity-purification assay. PCR products, which contained 0.0001% of the affinity-purified DNA obtained after each purification step, are shown in lanes 2-4. 15% of the PCR reaction products and 0.1% of the DNA input material were separated by agarose gel-electrophoresis. (B) Table describing the putative dSETDB1 target genes. Listed are genes and transposable elements, which associate with the MBDL of dSETDB1 *in vitro*. The table lists genes and transposable elements, the region of the genes and transposable elements, which were found to associate with dSETDB1 *in vitro*, and the corresponding reference sequences.
(1.01 MB EPS)

Figure S10 Functional characterization of the monoclonal antibody to dSETDB1 in Western Blot and immunoprecipitation (IP) assays. (A) Digital image of IP assays detecting dSETDB1 in total cell extracts prepared from S2 cells and nuclear extract prepared from 0-8 h old *Drosophila* embryos. Extracts were incubated with rat monoclonal antibody to dSETDB1. Protein-antibody complexes were precipitated using protein-G agarose, separated by SDS-PAGE, and electrophoretically transferred onto PVDF membrane. Western blots were developed using *anti*-dSETDB1 monoclonal rat antibody. Asterisks indicate the positions of the light and heavy chains of the *anti*-Flag antibody. (B) Digital image of Western blot analysis detecting dSETDB1 in total cell extracts prepared from *Sf*9 cells or *Sf*9 cells infected with recombinant baculovirus expressing Flag-epitope tagged dSETDB1 (Flag-dSETDB1). Cell extracts were separated by SDS-PAGE and electrophoretically transferred onto PVDF membrane. Western blots were developed using monoclonal *anti*-rat antibody to dSETDB1. (C) Digital image of Western blot analysis of IP assays detecting Flag-dSETDB1 using rat monoclonal antibody to dSETDB1. Flag-dSETDB1 was immunoprecipitated from total *Sf*9 extracts containing Flag-dSETDB1 using 1 µg dSETDB1 antibody and protein-G agarose beads (left) or Flag-beads containing 5–10 µg *anti*-Flag antibodies (right). Protein-antibody complexes were precipitated, separated by SDS-PAGE, and electrophoretically transferred onto PVDF membrane. Western blots were developed using rat monoclonal antibody to dSETDB1. (D) Digital image of Coomassie-Blue stained SDS-polyacrylamide gel detecting the presence of dSETDB1 in protein pools, which had been immunoprecipitated from nuclear extracts prepared from S2 cells and 0–8 h old embryos with antibody to dSETDB1. Immunoprecipitated proteins were separated by SDS-PAGE and detected by Coomassie Blue staining. Mass-spectrometry confirmed the presence of dSETDB1 in the protein bands marked with arrowheads.
(1.38 MB EPS)

Figure S11 DSETDB1 mediates repression of genes and retrotransposons. Schematic representation of Real-Time (RT) PCR assays corresponding to the Rvt-PCR assays shown in Figure 4A. RT-PCR assays were performed with the same cDNA pools used for conventional RvT-PCR. The level of transcription is presented in percent (%). The level of target gene transcription in S2 cells was set as 100%.
(0.27 MB EPS)

Figure S12 DSETDB1 does not control Dnmt2 and Su(var)205 transcription. Schematic representation of Real-Time (RT) PCR assays corresponding to the RvT-PCR assays shown in Figure 4A. RT-PCR assays were performed with the same cDNA pools used for conventional RvT-PCR. The level of transcription is presented in percent (%). The level of target gene transcription in S2 cells was set as 100%.
(0.25 MB EPS)

Figure S13 Functional characterization of the polyclonal antibody to ^5m^C. Autoradiogram of immunoprecipitation assays using rabbit serum or polyclonal antibody to ^5m^C. Antibodies were incubated with 0.1 µg [^32^P]-radiolabeled DNA oligonucleotides, which are not methylated (left) or contain three symmetrically methylated CpA-motifs (right). DNA-antibody complexes were precipitated using protein-A agarose. Retained DNA was purified, separated by native PAGE, and detected by autoradiography. The arrowhead marks the position of DNA oligonucleotides.
(0.52 MB EPS)

Figure S14 The *anti*-Dnmt2 polyclonal antibody detects Dnmt2 in Western Blot and immunoprecipitation (IP) assays. (A) Digital image of Western blot assays detecting Dnmt2 in total cell extracts prepared from *Sf*9 cells or *Sf*9 cells infected with recombinant baculovirus expressing Flag-epitope tagged Dnmt2. (B) Western blot analysis detecting Dnmt2 in total cell, extract prepared from S2 cells and nuclear extract prepared from 0–8 h old *Drosophila* embryos. (C) Western blot analyses of IP assays. 0.5 mg total S2 cell extract was incubated with rabbit serum or rabbit polyclonal antibody to Dnmt2. Protein-antibody complexes were precipitated with protein-A agarose. Cell extracts (A,B) and immunoprecipitated proteins (C) were separated by SDS-PAGE, electrophoretically transferred onto PVDF membrane, and developed using rabbit polyclonal antibody to Dnmt2 (A-C). Asterisks indicate the positions of the *anti*-Flag antibody light and heavy chains.
(1.38 MB EPS)

Figure S15 DSETDB1-mediated tri-methylation of H3-K9 mediates silencing and DNA methylation. Schematic representation of Real-Time PCR assays corresponding to the conventional PCR assays shown in Figure 4B. RT-PCR assays were performed using the same immunoprecipitated DNA pools used for conventional PCR. The degree of association of the antigens with the target DNA was calculated as fold enrichment by comparing the number of target DNA molecules in DNA pools obtained in ChIP assays using control antibodies with reactions containing antibodies to specific antigens.
(0.30 MB EPS)

Figure S16 The activities of the SET-domain and MBDL of dSETDB1 mediate initiation and spreading of DNA methylation at the *Rb* locus. Schematic representation of “bisulfite-treated DNA sequencing” assays. Genomic DNA was isolated from S2 cells transiently expressing GFP (mock) and S2 cells transiently co-expressing GFP and dSETDB1, dSETDB1(H775L), or dSETDB1(R436C). Genomic DNA was treated twice with bisulfite. The indicated regions of the PDE and Exon-I of *Rb* were amplified by PCR and cloned into pCR2.1-TOPO. 10 PCR products were sequenced for each bisulfite reaction. The y-axis shows the CpN methylation rate in percent (%) for regions within the PDE (left) and the Exon-I (right) of *Rb*. The CpN methylation rate was calculated by dividing the number of methylation events at CpN-motifs by the total number of CpN-motifs present in tested DNA fragments. The shown data represents the mean value of the CpN methylation rates obtained form a total of 20 clones generated in two different “bisulfite-treated DNA sequencing” assays. Error bars represent the standard error of the mean (SEM).
(2.58 MB EPS)

Figure S17 DSETDB1 mediates DNA methylation at the *Antp* and *CG2316* and *Rt1b{}799* loci. Schematic representation of “bisulfite-treated DNA sequencing” assays. Genomic DNA was isolated from S2 cells transiently expressing GFP (mock) and S2 cells transiently co-expressing GFP and dSETDB1, dSETDB1(H775L), or dSETDB1(R436C). Bisulfite-assays were performed and analyzed as described in Figure S16 except that DNA methylation was monitored at DNA fragments corresponding to the enhancer region of *Antp* and *CG2316* and *Rt1b{}799*.
(3.61 MB EPS)

Figure S18 DSETDB1 controls initiation and spreading of DNA methylation on the *Rb* locus. Schematic representation of Real-Time PCR assays corresponding to the conventional PCR assays shown in Figure 5A. RT-PCR assays were performed using the same immunoprecipitated DNA pools used for conventional PCR. The association of the antigens with the target DNA was calculated as fold enrichment by comparing the number of target DNA molecules in DNA pools obtained in ChIP assays using control antibodies with reactions containing antibodies to specific antigens.
(0.31 MB EPS)

Figure S19 DSETDB1 preferentially tri-methylates H3-K9 at target genes. Digital images of ethidium bromide-stained agarose gel showing the PCR products for the PDE of *Rb* (see Figure 5) and the promoter of the *tetO-tk-luc* reporter gene in DNA pools obtained by ChIP. Chromatin was isolated from S2 cells (top) and *tetO-tk-luc S2* cells (bottom) transiently expressing dSETDB1. Chromatin was immunoprecipitated with antibodies to mono-methylated H3-K9, di-methylated H3-K9, and tri-methylated H3-K9 or rabbit serum (mock). PCR detected the presence of the PPE in immunoprecipitated DNA pools. Input represents the amount of target DNA present in 1% of the chromatin used for ChIP.
(0.53 MB EPS)

Figure S20 The MBDL of DSETDB1 is involved in silencing. Schematic representation of Real-Time PCR assays corresponding to the conventional PCR assays shown in Figure 5B. RT-PCR assays were performed using the same immunoprecipitated DNA pools used for conventional PCR. The degree of association of the antigens with the target DNA was calculated as fold enrichment by comparing the number of target DNA molecules in DNA pools obtained in ChIP assays using control antibodies with reactions containing antibodies to specific antigens.
(0.26 MB EPS)

Figure S21 DSETDB1 mediates methylation at the *Rb* locus. Schematic representation of “bisulfite-treated DNA sequencing” assays. Genomic DNA was isolated from S2 cells transiently expressing GFP (mock), and S2 cells transiently co-expressing GFP and dSETDB1, dSETDB1(H775L), or dSETDB1(R436C). Genomic DNA was treated twice with bisulfite. The indicated regions of the PDE and Exon-I of Rb were amplified by PCR and cloned into pCR2.1-TOPO. 10 PCR products were sequenced for each bisulfite reaction. The grey boxes indicate the number of detected methylation events at individual CpN-motifs present in a highly methylated region within the PDE (left) and Exon-I (right) of Rb. DSETDB1 mediates methylation at the Rb locus. Schematic representation of “bisulfite-treated DNA sequencing” assays. Genomic DNA was isolated from S2 cells transiently expressing GFP (mock), and S2 cells transiently co-expressing GFP and dSETDB1, dSETDB1(H775L), or dSETDB1(R436C). Genomic DNA was treated twice with bisulfite. The indicated regions of the PDE and Exon-I of Rb were amplified by PCR and cloned into pCR2.1-TOPO. 10 PCR products were sequenced for each bisulfite reaction. The grey boxes indicate the number of detected methylation events at individual CpN-motifs present in a highly methylated region within the PDE (left) and Exon-I (right) of *Rb*.
(0.45 MB EPS)

Figure S22 Dnmt2 and Su(var)205 associate *in vitro* and in *Drosophila*. (A,B) Fluorograms of *in vitro* protein-protein interaction assays programmed with Flag-beads loaded with *Sf*9 cell extract (control) or recombinant, Flag-epitope tagged dSETDB1, Dnmt2, and Su(var)205. Protein-loaded Flag-beads were incubated with *in vitro* translated, [^35^S]-methionine labeled (A) Dnmt2 or (B) Su(var)205. “Input” represents 5% of the input material used in binding assays (C,D) Western blot analysis of immunoprecipitation assays detecting the association of Dnmt2 and Su(var)205 in total cell extracts prepared from 0-8 h old *Drosophila* embryos. Extracts were incubated with antibodies to dSETDB1, Dnmt2, and Su(var)205. Precipitated proteins were separated by SDS-PAGE, electrophoretically transferred onto PVDF-membrane, and developed using antibodies to (C) Dnmt2 and (D) Su(var)205.
(2.25 MB EPS)

Figure S23 Knockdown of Dnmt2 and Su(var)205 through RNAi. (A,B) Digital images of Western blot assays using total cell extract isolated from (A-C) S2 cells treated with control siRNA, which targets human GAPDH (mock-RNAi); (A) S2 cells treated with siRNA Dnmt2(1) [Dnmt2(1)-RNAi] or siRNA Dnmt2(2) [Dnmt2(2)-siRNA], which target the Dnmt2 mRNA. Extracts were separated by SDS-PAGE, electrophoretically transferred onto PVDF membrane, and developed with rabbit monoclonal antibody to Dnmt2. (B,C) S2 cells were treated with siRNA Su(var)205(1) [Su(var)205(1)-RNAi] or siRNA Su(var)205(2) [Su(var)205(2)-siRNA], which target the Su(var)205 mRNA. Extracts were prepared using denaturing buffer containing 8M urea (B) or PBS (C), separated by SDS-PAGE, electrophoretically transferred onto PVDF membrane, and developed with rabbit monoclonal antibody to Su(var)205. Note that Su(var)205 migrates as a 40 KD protein band in the absence of urea (C).
(1.40 MB EPS)

Figure S24 Dnmt2 and Su(var)205 regulate *Rb* transcription. Schematic representation of Real-Time (RT) PCR assays corresponding to the Rvt-PCR assays shown in Figure 6A,B. RT-PCR assays were performed with the same cDNA pools used for conventional RvT-PCR. The level of transcription is presented in percent (%). The level of target gene transcription in S2 cells was set as 100%.
(0.24 MB EPS)

Figure S25 Dnmt2 and Su(var)205 regulate the transcription of genes and retrotransposons. Schematic representation of Real-Time (RT) PCR assays corresponding to the RvT-PCR assays shown in Figure 7A. RT-PCR assays were performed with the same cDNA pools used for conventional RvT-PCR. The level of transcription is presented in percent (%). The level of target gene transcription in S2 cells was set as 100%.
(0.29 MB EPS)

Figure S26 Su(var)205 and Dnmt2 mediate DNA methylation of *Rb*. Schematic representation of Real-Time PCR assays corresponding to the conventional PCR assays shown in Figure 6C. RT-PCR assays were performed using the same immunoprecipitated DNA pools used for conventional PCR. The degree of association of the antigens with the target DNA was calculated as fold enrichment by comparing the number of target DNA molecules in DNA pools obtained in ChIP assays using control antibodies with reactions containing antibodies to specific antigens.
(0.28 MB EPS)

Figure S27 Dnmt2 and Su(var)205 mediate spreading of DNA methylation on the *Rb* locus. Digital images of ethidium bromide-stained agarose gels showing the PCR product for the Exon-I fragment of *Rb* (Fig. 5C) in DNA pools obtained by ChIP. The DNA pools used for the PCR assays are the same DNA pools, which were used to detect the PDE of *Rb* (Fig. 5A). Chromatin was isolated from S2 cells which did (+) or did not (-) transiently express dSETDB1, and were treated with control siRNA, which targets human GAPDH (mock-RNAi); (left) S2 cells treated with siRNA Dnmt2(1) (Dnmt2-RNAi), which targets the Dnmt2 mRNA; and (right) S2 cells treated with siRNA (Su(var)205-RNAi), which targets the Su(var)205 mRNA. Chromatin was immunoprecipitated with antibodies to dSETDB1, Dnmt2, Su(var)205, or ^5m^C. Input represents the amount of PCR product for Exon-I of *Rb* detectable in 3% of the chromatin sample used in immunoprecipitation assays.
(5.11 MB EPS)

Figure S28 Dnmt2-mediated DNA methylation at the *Rb* and *Antp* loci. Schematic representations of “bisulfite-treated DNA sequencing” assays. Genomic DNA was isolated from S2 cells incubated with siRNA targeting human GAPDH (mock) or siRNA targeting Dnmt2 mRNA. Bisulfite-assays were performed and analyzed as described in Figure S21 except that DNA methylation was monitored at DNA fragments corresponding to the PDE of *Rb* and the enhancer region of *Antp*.
(0.44 MB EPS)

Figure S29 Dnmt2 mediates DNA methylation at genes and *Rt1b* retrotransposons. Schematic representation of Real-Time PCR assays corresponding to the conventional PCR assays shown in Figure 7B. RT-PCR assays were performed using the same immunoprecipitated DNA pools used for conventional PCR. The degree of association of the antigens with the target DNA was calculated as fold enrichment by comparing the number of target DNA molecules in DNA pools obtained in ChIP assays using control antibodies with reactions containing antibodies to specific antigens.
(0.28 MB EPS)

Figure S30 Dnmt2-mediated DNA methylation at the *CG2316* and *Rt1b{}799* loci. Schematic representations of “bisulfite-treated DNA sequencing” assays. Genomic DNA was isolated from S2 cells incubated with siRNA targeting human GAPDH (mock) or siRNA targeting Dnmt2 mRNA. Bisulfite-assays were performed and analyzed as described in Figure S21 except that DNA methylation was monitored at DNA fragments corresponding to *CG2316* and *Rt1b{}799*.
(0.45 MB EPS)

Figure S31 Su(var)205 regulates DNA methylation at genes and retrotransposons. Schematic representation of RT-PCR assays corresponding to the conventional PCR assays shown in Figure 7C. The same immunoprecipitated DNA pools used for conventional PCR and RT-PCR. The degree of association of the antigens with the target DNA was calculated as fold enrichment by comparing the number of target DNA molecules in DNA pools obtained in ChIP assays using control antibodies with reactions containing antibodies to specific antigens.
(0.28 MB EPS)

Figure S32 Knockdown of dSETDB1 expression through RNA interference (RNAi). (A) Digital image of Western blot assays of immunoprecipitation assays using whole protein extract prepared from 0.2 g 0–8 h old embryos and 1,000 eye imaginal discs containing the indicated Gal4 driver and Gal4-dependent reporter genes. The *actin5C^Gal4^* driver strain (*Act5C^Gal4^*) expresses Gal4 ubiquitously in *Drosophila* embryos. The *lozenge* (*lz*) Gal4 driver (*lzGal4*) expresses Gal4 in cells posterior and “to a lesser extent” anterior to the morphogenetic furrow in developing eye imaginal discs. The Gal4-dependent reporter *UAS-dSETDB1.IR*, which transcribes a dsRNA targeting the dSETDB1 mRNA. Total protein extracts were incubated with rat monoclonal antibody to dSETDB1. Protein-antibody complexes were precipitated with protein-G agarose, separated by SDS-PAGE, electrophoretically transferred onto PVDF membrane, and analyzed by Western blot using antibody to dSETDB1. The asterisk indicates the position of the heavy chain of the dSETDB1 antibody. The positions and relative molecular weights (rMW) of protein standards are indicated to the left. (B) Digital images of immunostaining assays detecting dSETDB1 and histone H3 phosphorylated at serine 10 [phospho-H3(Ser10)], which is a marker of mitosis, in eye imaginal discs isolated from third instar larvae containing the Gal4 driver and reporter constructs described in (A). Eye imaginal discs were isolated from third instar larvae and incubated with rat monoclonal antibody to dSETDB1 and rabbit polyclonal antibody to phospho-H3(Ser10). DSETDB1 (purple/brown) was detected using *anti*-rat secondary antibody coupled to alkaline phosphatase and the “Red Alkaline Phosphatase Substrate kit” (Vector Laboratories). Phospho-H3(Ser10) (dark brown) was detected using an *anti*-rabbit secondary antibody coupled to horseradish peroxidase and diaminobenzidine and peroxidae as substrates. The arrowhead marks the position of the morphogenetic furrow (MF). The enhanced staining on the right site of the eye imaginal discs results from folding of the eye discs.
(1.60 MB EPS)

Figure S33 DSETDB1 represses *PCNA* transcription. Schematic representation of Real-Time (RT) PCR assays monitoring *Rb* and *PCNA* transcription in posterior and anterior halves of eye imaginal discs. RNA pools were isolated from posterior and anterior halves of eye imaginal discs, which were isolated from 3^rd^ instar larvae of the genotypes described in Figure 8. Discs were separated at the morphogenetic furrow. RNA was reverse transcribed and the resulting cDNA pools served as a template for RT-PCR assays monitoring *Rb* (A) and *PCNA* (B) transcription. The level of transcription is presented in percent (%). The level of target gene transcription in eye imaginal discs isolated from *lz^Gal4,^* larvae was set to 100%.
(0.25 MB EPS)

Figure S34 DSETDB1 mediates methylation and silencing of *Rb* in the developing eye. Schematic representation of Real-Time PCR assays corresponding to the conventional PCR assays shown in Figure 9C. RT-PCR assays were performed using the same immunoprecipitated DNA pools used for conventional PCR. The degree of association of the antigens with the target DNA was calculated as fold enrichment by comparing the number of target DNA molecules in DNA pools obtained in ChIP assays using control antibodies with reactions containing antibodies to specific antigens.
(0.26 MB EPS)

Figure S35 DSETDB1 silences the transcription of *Rt1b{}* and *HeT-A* retrotransposons. Schematic representation of Real-Time (RT) PCR assays corresponding to the RvT-PCR assays shown in Figure 10B,C. RT-PCR assays were performed with the same cDNA pools used for conventional RvT-PCR. The level of transcription is presented in percent (%). The level of target gene transcription in imaginal discs isolated from *Gal4(71)* larvae was set as 100%.
(0.25 MB EPS)

Figure S36 DSETDB1 mediates methylation and silencing of *Rt1b{}* and *HeT-A* retrotransposons Schematic representation of Real-Time PCR assays corresponding to the conventional PCR assays shown in Figure 10D,E. RT-PCR assays were performed using the same immunoprecipitated DNA pools used for conventional PCR. The degree of association of the antigens with the target DNA was calculated as fold enrichment by comparing the number of target DNA molecules in DNA pools obtained in ChIP assays using control antibodies with reactions containing antibodies to specific antigens.
(0.29 MB EPS)

Figure S37 Dnmt2 mediates DNA methylation of *Rt1b{}* and *HeT-A* retrotransposons in the developing wing. Schematic representations of “bisulfite-treated DNA sequencing” assays. Genomic DNA was isolated from 50 wing imaginal discs of 3^rd^ instar larvae, which lack dSETDB1 [*Gal4(71B);UAS-dSETDB1.IR*] or Dnmt2 [*Gal4(71B);UAS-Dnmt2*] through RNAi or control larvae (*UAS-dSETDB1.IR* and *UAS-Dnmt2*). Genomic DNA was treated twice with bisulfite. DNA fragments containing the depicted DNA sequences were amplified by PCR and cloned into pCR2.1-TOPO. 10 PCR products were sequenced for each bisulfite reaction. The grey boxes indicate the number of detected methylation events at individual CpN-motifs present in a highly methylated region within the *Rt1b{}* (left) and *HeT-A* (right) retrotransposons.
(0.46 MB EPS)

Table S1 DNA oligonucleotides used for PCR and RvT-PCR.
(0.12 MB DOC)

Table S2 DNA oligonucleotides used for DNA-protein interaction assays.
(0.05 MB DOC)

## References

[1] Bird AP, Wolffe AP (1999). Methylation-induced repression – belts, braces, and chromatin.. Cell.

[2] Wilson GG, Murray NE (1991). Restriction and modification systems.. Annu Rev Genet.

[3] Jaenisch R, Bird A (2003). Epigenetic regulation of gene expression: how the genome integrates intrinsic and environmental signals.. Nat Genet.

[4] Suzuki MM, Bird A (2008). DNA methylation landscapes: provocative insights from epigenomics.. Nat Rev Genet.

[5] Klose RJ, Bird AP (2006). Genomic DNA methylation: the mark and its mediators.. Trends Biochem Sci.

[6] Chan SW, Henderson IR, Jacobsen SE (2005). Gardening the genome: DNA methylation in Arabidopsis thaliana.. Nat Rev Genet.

[7] Lyko F, Beisel C, Marhold J, Paro R (2006). Epigenetic regulation in *Drosophila*.. Curr Top Microbiol Immunol.

[8] Goll MG, Kirpekar F, Maggert KA, Yoder JA, Hsieh CL (2006). Methylation of tRNAAsp by the DNA methyltransferase homolog Dnmt2.. Science.

[9] Kunert N, Marhold J, Stanke J, Stach D, Lyko F (2003). A Dnmt2-like protein mediates DNA methylation in *Drosophila*.. Development.

[10] Phalke S, Nickel O, Walluscheck D, Hortig F, Onorati MC (2009). Retrotransposon silencing and telomere integrity in somatic cells of *Drosophila* depends on the cytosine-5 methyltransferase DNMT2.. Nat Genet.

[11] Stabell M, Bjorkmo M, Aalen RB, Lambertsson A (2006). The SET domain encoding gene dEset is essential for proper development.. Hereditas.

[12] Clough E, Moon W, Wang S, Smith K, Hazelrigg T (2007). Histone methylation is required for oogenesis in.. Development.

[13] Seum C, Reo E, Peng H, Rauscher FJ, Spierer P (2007). SETDB1 is required for chromosome 4 silencing.. PloS Genet.

[14] Tzeng TY, Lee CH, Chan LW, Chen CK (2007). Epigenetic regulation of the chromosome 4 by the histone H3K9 methyltransferase dSETDB1.. Pro Natl Acad Sci USA.

[15] Bird A (2002). DNA methylation patterns and epigenetic memory.. Genes Dev.

[16] Ehrlich M, Gama-Sosa MA, Huang LH, Midgett RM, Kuo KC (1982). Amount and distribution of 5-methylcytosine in human DNA from different types of tissues of cells.. Nucleic Acids Res.

[17] Gowher H, Leismann O, Jeltsch A (2000). DNA of *Drosophila melanogaster* contains 5-methylcytosine.. EMBO J.

[18] Lyko F, Ramsahoye BH, Jaenisch R (2000). DNA methylation in *Drosophila melanogaster*.. Nature.

[19] Salzberg A, Fisher O, Siman-Tov R, Ankri S (2004). Identification of methylated sequences in genomic DNA of adult *Drosophila melanogaster*.. Biochem Biophys Res Commun.

[20] Jackson JP, Lindroth AM, Cao X, Jacobsen SE (2002). Control of CpNpG DNA methylation by the KRYPTONITE histone H3 methyltransferase.. Nature.

[21] Lehnertz B, Ueda Y, Derijck AA, Braunschweig U, Perez-Burgos L (2003). Suv39h-mediated histone H3 lysine 9 methylation directs DNA methylation to major satellite repeats at pericentric heterochromatin.. Curr Biol.

[22] Tamaru H, Selker EU (2001). A histone H3 methyltransferase controls DNA methylation in *Neurospora crassa*.. Nature.

[23] Viré E, Brenner C, Deplus R, Blanchon L, Fraga M (2006). The Polycomb group protein EZH2 directly controls DNA methylation.. Nature.

[24] Jones PA, Baylin SB (2007). The epigenomics of cancer.. Cell.

[25] Monk M, Boubelik M, Lehnert S (1987). Temporal and regional changes in DNA methylation in the embryonic, extraembryonic and germ cell lineages during mouse embryo development.. Development.

[26] Eckhardt F, Lewin J, Cortese R, Rakyan VK, Attwood J (2006). DNA methylation profiling of human chromosomes 6, 20 and 22.. Nat Genet.

[27] Henderson IR, Jacobsen SE (2007). Epigenetic inheritance in plants.. Nature.

[28] Illingworth R, Kerr A, Desousa D, Jørgensen H, Ellis P (2008). A novel CpG island set identifies tissue-specific methylation at developmental gene loci.. PLoS Biol.

[29] Vaughn MW, Tanurdzic M, Lippman Z, Jiang H, Carrasquillo R (2007). Epigenetic natural variation in *Arabidopsis thaliana*.. PLoS Biol.

[30] Weber M, Davies JJ, Wittig D, Oakeley EJ, Haase M (2005). Chromosome-wide and promoterspecific analyses identify sites of differential DNA methylation in normal and transformed human cells.. Nat Genet.

[31] Zilberman D, Gehring M, Tran RK, Ballinger T, Henikoff S (2007). Genome-wide analysis of *Arabidopsis thaliana* DNA methylation uncovers an interdependence between methylation and transcription.. Nat Genet.

[32] Hellman A, Chess A (2007). Gene body-specific methylation on the active X chromosome.. Science.

[33] Brower-Toland B, Riddle NC, Jiang H, Huisinga KL, Elgin SCR (2009). Multiple SET methyltransferases are required to maintain normal heterochromatin domains in the genome of *Drosophila melanogaster*.. Genetics.

[34] Richards EJ, Elgin SCR (2002). Epigenetic codes for heterochromatin formation and silencing: rounding up the usual suspects.. Cell.

[35] Baron U, Goshen M, Bujard H (1997). Tetracycline controlled transcription in eukaryotes: novel transactivators with graded transactivation potential.. Nucl Acids Res.

[36] Hendrich B, Tweedie S (2003). The methyl-CpG binding domain and the evolving role of DNA methylation in animals.. Trends Genet.

[37] Nan X, Meehan RR, Bird AP (1993). Dissection of the methyl-CpG binding domain from the chromosomal protein MeCP2.. Nucleic Acids Res.

[38] Kaminker JS, Bergman CM, Kronmiller B, Carlson J, Svirskas R (2002). The transposable elements of the Drosophila melanogaster euchromatin: a genomics perspective.. Genome Biol.

[39] Du W, Vidal M, Xie JE, Dyson N (1996). *RBF*, a novel *RB*-related gene that regulates E2F activity and interacts with cyclin E in *Drosophila*.. Genes Dev.

[40] Hallstrom TC, Nevins JR (2009). Balancing the decision of cell proliferation and cell fate.. Cell Cycle.

[41] Ferres-Marco D, Gutierrez-Garcia I, Vallejo DM, Bolivar J, Gutierrez-Aviño FJ (2006). Epigenetic silencers and Notch collaborate to promote malignant tumours by *Rb* silencing.. Nature.

[42] Morata G (1993). Homeotic genes of *Drosophila*.. Curr Opin Genet Dev.

[43] Ryder E, Blows F, Ashburner M, Bautista-Llacer R, Coulson D (2004). The DrosDel collection: a set of P-element insertions for generating custom chromosomal aberrations in *Drosophila melanogaster*.. Genetics.

[44] Narsa Reddy M, Tang LY, Lee TL, James Shen CK (2003). A candidate gene for *Drosophila* genome methylation.. Oncogene.

[45] Smallwood A, Estève PO, Pradhan S, Carey M (2007). Functional cooperation between HP1 and DNMT1 mediates gene silencing.. Genes Dev.

[46] Keller SA, Ullah Z, Buckley MS, Henry RW, Arnosti DN (2005). Distinct developmental expression of *Drosophila* retinoblastoma factors.. Gene Expr Patterns.

[47] Xin S, Weng L, Xu J, Du W (2002). The role of *RB*F in developmentally regulated cell proliferation in the eye disc and in Cyclin D/Cdk4 induced cellular growth.. Development.

[48] Zemach A, Grafi G (2007). Methyl-CpG-binding domain proteins in plants: interpreters of DNA methylation.. Trends Plant Sci.

[49] Zhang X, Yazaki J, Sundaresan A, Cokus S, Chan SW (2006). Genome-wide high-resolution mapping and functional analysis of DNA methylation in *Arabidopsis*.. Cell.

[50] Hark AT, Schoenherr CJ, Katz DJ, Ingram RS, Levorse JM (2000). CTCF mediates methylation-sensitive enhancer-blocking activity at the H19/Igf2 locus.. Nature.

[51] Rountree MR, Selker EU (1997). DNA methylation inhibits elongation but not initiation of transcription in *Neurospora crassa*.. Genes Dev.

[52] Blomen VA, Boonstra J (2007). Cell fate determination during G1 phase progression.. Cell Mol Life Sci.

[53] Baylin SB (2005). DNA methylation and gene silencing in cancer.. Nat Clin Pract Oncol.

[54] Keshet I, Schlesinger Y, Farkash S, Ran E, Hecht M (2006). Evidence for an instructive mechanism of methylation in cancer cells.. Nat Genet.

[55] Grønbaek K, Hother C, Jones PA (2007). Epigenetic changes in cancer.. APMIS.

[56] Maile T, Kwoczynski S, Katzenberger RJ, Wassarman DA, Sauer F (2004). TAF1 activates transcription by phosphorylation of serine 33 in histone H2B.. Science.

[57] Yuan B, Latek R, Hossbach M, Tuschl T, Lewitte F (2004). siRNA Selection Server: an automated siRNA oligonucleotide prediction server.. Nucleic Acids Res.

[58] Crew JR, Batterham P, Pollock JA (1997). Developing compound eye in lozenge mutants of *Drosophila*: lozenge expression in the R7 equivalence group.. Dev Genes Evol.

[59] Brand A, Perrimon N (1993). Targeted gene expression as a means of altering cell fates and generating dominant phenotypes.. Development.

[60] Ashburner M, Golic KG, Hawley RS (2005). *Drosophila*: A Laboratory Handbook..

